# A Novel Cuprotosis-Related Gene FDX1 Signature for Overall Survival Prediction in Clear Cell Renal Cell Carcinoma Patients

**DOI:** 10.1155/2022/9196540

**Published:** 2022-09-05

**Authors:** Wei-Tong Zhang, Yi-Ming Gong, Chao-yang Zhang, Jia-shan Pan, Tao Huang, Yong-Xiang Li

**Affiliations:** ^1^Department of General Surgery, The First Affiliated Hospital of Anhui Medical University, Hefei 230022, China; ^2^Urology Department, The First Affiliated Hospital of University of Science and Technology of China, Hefei 230022, China; ^3^Urology Department, The First Affiliated Hospital of Anhui Medical University, Hefei 230022, China

## Abstract

**Background:**

Ferredoxin 1 (FDX1) is a newly discovered gene regulating cuprotosis. However, the effect of FDX1 expression on clear renal cell carcinoma (ccRCC) is unknown.

**Methods:**

Gene expression profiles and clinical data of ccRCC patients were downloaded from the Cancer Genome Atlas (TCGA) database. The differences in FDX1 expression between ccRCC and nonneoplastic tissues adjacent to cancer were analyzed by R software. The results were validated by GEO data, quantitative real-time polymerase chain reaction (qRT-PCR), western blotting (WB), and immunohistochemistry (IHC). Chi-square test was used to analyze the clinical pathological parameters. Kaplan-Meier survival analysis and Cox proportional hazard regression model selection were used to evaluate the effect of FDX1 expression on overall survival. Protein interaction networks were used to analyze other proteins that interact with FDX1. Signal pathway analysis was performed for possible FDX1 enrichment using GSEA and ssGSEA algorithms. Pan-cancer analysis of FDX1 was carried out through TCGA database.

**Results:**

The FDX1 expression in nontumor tissues was significantly higher than that in ccRCC, and the expression difference was verified by GEO data, qRT-PCR, WB, and IHC. The high expression of FDX1 was significantly related to the well overall survival rate (*P* < 0.05). The chi-square test showed that the high expression of FDX1 was related to gender, TNM stage, T stage, lymph node metastasis, and pathological grade. Additionally, the FDX1 expression level was different in groups classified based on pathological grade, gender, TNM stage, T stage, lymph node metastasis, and distant metastasis (*P* < 0.05). The multivariate analysis revealed the high expression of FDX1 as an important independent predictor for overall survival. STRING database results showed that LIAS and LIPT1 may interact with FDX1 in the PPI network, which are also involved in the regulation of cuprotosis. The GSEA and ssGSEA results showed that the FDX1 was enriched in the anticancer pathway. The FDX1 high expression is associated with better prognosis in many cancers, as revealed by pan-cancer analysis.

**Conclusion:**

FDX1 may play a role in the progression of ccRCC as a tumor suppressor gene. It can be used as a potential prognostic indicator and therapeutic target of ccRCC. However, the cuprotosis regulatory role in the development of ccRCC needs to be further verified.

## 1. Introduction

Renal cell carcinoma (RCC) accounts for about 2% of overall cancer diagnoses and deaths worldwide [1]. The majority of renal cancer patients have clear renal cell carcinoma (ccRCC), accounting for 70%–80% [2]. The treatment of ccRCC is mainly surgical. Moreover, it is not sensitive to chemotherapy and radiotherapy. Compared with other pathological types, patients with ccRCC have a worse prognosis and are more prone to metastasis in distant organs such as the lungs and bone [3]. Therefore, establishing effective prognostic biomarkers is essential for accurate prognosis and rationalized treatment strategies in ccRCC patients.

In recent years, researchers have studied the cell death mechanism extensively, which is an inevitable and complicated process. Nonetheless, there are multiple pathways for cell death induction. In the 1960s, researchers realized that molecular mechanisms could regulate cell death, help in normal physiological functions, and lead to pathological changes. Hence, the concept of “programmed cell death” was proposed [4]. Ferroptosis is a type of iron-dependent programmed cell death discovered by Brent R. Stockwell Laboratory of Columbia University in 2012 [5]. Ferroptosis is induced by the excessive accumulation of lipid peroxide. Notably, its morphological characteristics, mode of action, and molecular mechanism are completely different from other programmed cell deaths [6]. In recent years, it has garnered the attention of scholars worldwide. It has been found that ferroptosis is related to various tumors [7–9]. As renal cancers are mostly resistant to chemotherapy and radiotherapy, regulatory cell death is an ideal treatment strategy for ccRCC, which may help to overcome the drug resistance in ccRCC [10].

The concept of cuprotosis was first proposed in a paper published on Science on 17 March 2022 [11]. Like iron, copper is also a basic element for life activities in all living beings. As a necessary auxiliary factor of enzymes, copper plays an essential role in life activities. Copper is a trace element in the human body. An active steady-state mechanism maintains the concentration of intracellular copper ions at a very low level. However, once the threshold is exceeded, copper becomes toxic, leading to cell death. Besides, the mechanism of cuprotosis was not clear. This study has confirmed that the copper-dependent controlled cell death mode is a new cell death mode different from the already known cell death mechanism [11]. A copper ion can still induce cell death despite inhibiting the known cell death modes. However, whether cuprotosis affects the progression of tumors like ferroptosis is not known. Additionally, the FDX1 gene is essential for copper-induced cell death [11]. Therefore, we studied the FDX1 expression in ccRCC and its correlation with the prognosis of these patients. In this study, we collected mRNA expression data from published TCGA data to study the clinical relationship between FDX1 and ccRCC. At the same time, we verified the expression of FDX1 in GEO data, qRT-PCR, WB, and IHC.

## 2. Materials and Methods

### 2.1. Data Acquisition

The original messenger RNA gene data of 541 ccRCC tissues and 72 nontumor tissues were downloaded from TCGA database (https://portal.gdc.cancer.gov) on or before April 10, 2022. In addition, clinical data of ccRCC patients were also obtained from TCGA database (Table 1).

### 2.2. Verification of FDX1 Expression by the GEO Database

In the NCBI (https://www.ncbi.nlm.nih.Gov/), GEO datasets were searched for “clear cell renal cell carcinoma” in *Homo sapiens*. Two datasets (GSE53757 and GSE40435) were downloaded, including 173 ccRCC tissues and 173 adjacent nontumor tissues (Table 2). GEO data was used to verify the differences in FDX1 expression between these two tissue types.

### 2.3. Verification of FDX1 Expression by qRT-PCR, WB, and IHC

Total RNA was extracted from 20 pairs of ccRCC tissues and adjacent nontumor tissues by TRIzol reagent (Invitrogen). A UV spectrophotometer was used to determine the concentration and purity of RNA. cDNA was synthesized by reverse transcriptase and amplified. Each sample was measured in triplicate. The PCR primers used for amplification were as follows: FDX1, 5′-TTCAACCTGTCACCTCATCTTTG-3′ (forward), 5′-TGCCAGATCGAGCATGTCATT-3′ (reverse); GAPDH as an endogenous control, 5′ATCAAGAAGGTGGTGAAGCAGG-3′ (forward), 5′-CGTCAAAGGTGGAGGAGTGG-3′ (reverse). The relative expression levels of FDX1 were calculated using the 2 − ΔΔCT method.

Total protein was extracted from 16 pairs of fresh tissues preserved in liquid nitrogen. The total protein concentration was determined by a BCA protein concentration determination kit. 10 *μ*g of each sample was used for electrophoresis. The separated proteins were transferred onto the membrane and blocked in 5% skim milk powder. The membrane was incubated overnight in a hybridization bag filled with diluted primary antibody working solution of FDX1 (1 : 1000, cat 12592-1-AP, Proteintech). The membrane was washed with PBS three times for 15 minutes each. The secondary antibody was incubated at room temperature for 2 h and exposed, and the results were observed.

Five pairs of tissues were embedded and presectioned. Paraffin sections were deparaffinized and hydrated through water; endogenous peroxidase was blocked by 3% H_2_O_2_; after washing with PBS, EDTA solution was repaired by a microwave for 6 min, and the first antibody was added dropwise at 37°C for incubation for 1 h; after washing with PBS, the second antibody labeled with peroxidase was added dropwise and incubated at 37°C for 45 min. Color was developed with a DAB chromogenic solution. Then the slices were stained with hematoxylin, dehydrated, transparentized, and sealed using neutral gum. PBS was used instead of primary antibody as negative control. FDX1 is positively stained with the presence of yellowish-brown fine particles in the cytoplasm of the cells.

### 2.4. FDX1 Expression Analysis and Survival Analysis

FDX1 mRNA expression levels were divided into two groups (high FDX1 expression and low FDX1 expression group) based on a median expression. The Kaplan-Meier survival curve was obtained by visualizing the survival software package of R software.

### 2.5. Univariate and Multivariate Cox Analyses

Cox proportional hazard regression model was used for univariate and multivariate analysis. Risk ratios and 95% confidence intervals were calculated to quantitatively assess independent predictors of survival by clinical pathology parameters and FDX1 expression.

### 2.6. Protein Human Expression Atlas Database

The HPA database (Human Protein Atlas) contains proteomics, transcriptomics, and systems biology data on protein expression in normal and cancerous tissues. HPA was used to analyze the differential expression of proteins in normal and tumor tissues.

### 2.7. STRING Database

This database is a search tool for analyzing the interaction of biological genes or proteins. “FDX1” was input, the human was selected as the species type, medium 0.4 was selected as the confidence level, and 20 was selected as the maximum number of interactions for searching in the STRING database.

### 2.8. Gene Set Enrichment Analysis

GSEA is a computational method that can enrich genes in signal pathways. In this study, GSEA generated an ordered matrix according to the correlation between all genes with the expression of FDX1 and divided it into two groups (high FDX1 expression and low FDX1 expression group) based on the median expression. After GSEA, the signal pathways enriched in the high and low groups of FDX1 were obtained. Each analysis was performed for 1000 genome randomizations. First, the gene set contained in the related pathways was collected. Then, the enrichment score of each sample in each pathway was sequentially calculated according to the ssGSEA algorithm to obtain the association between the sample and the pathway. Finally, the relationship between the gene and the pathway was obtained by calculating the correlation between the gene expression and the pathway score [12].

### 2.9. Analysis of FDX1 in Pan-Cancer

Expression data and corresponding clinical information on tumors were obtained from TCGA database. The univariate Cox regression analysis and “forest plot” R package were used to show the *P* value, HR, and 95% CI.

### 2.10. Statistical Analysis

Mann–Whitney *U* test was used to analyze the expression difference of FDX1 between ccRCC tissue and adjacent nontumor tissues. Chi-square (*χ*^2^) test was used to evaluate the FDX1 expression relationship with clinicopathological parameters. Kaplan-Meier analysis and logarithmic rank test were used to compare the survival rate between the high and low expression group of FDX1. Cox proportional hazard regression model was used for single- and multifactor survival analysis. SPSS software (version 23.0) and R software (version 4.20) were used for all statistical analyses. The significance level was determined with *P* < 0.05. We followed the methods of Chen et al. [13].

## 3. Results

### 3.1. The Difference in FDX1 Expression in ccRCC Based on TCGA Data

The mRNA level obtained from TCGA database showed that FDX1 in normal tissues adjacent to cancer was higher than in the cancer tissues. The scatter plots show the mRNA expression of FDX1 in ccRCC tissues and adjacent nonneoplastic tissues (*P* < 0.05) (Figure 1(a)).

### 3.2. Verification of the Difference in FDX1 Expression in ccRCC Based on GEO Data

The expression difference of FDX1 was verified in GSE53757 and GSE4043 data for 173 ccRCC tissues and 173 adjacent nontumor tissue samples, respectively (Table 2). In both groups, the expression of FDX1 in adjacent nonneoplastic tissues to ccRCC tissues was higher than in cancer tissues (*P* < 0.05) (Figures 1(b) and 1(c)).

### 3.3. Verify the Difference in FDX1 Expression in ccRCC by qRT-PCR, WB, and IHC

We used qRT-PCR to evaluate the FDX1 expression at the transcription level. We found that in 20 pairs of ccRCC and adjacent nontumor tissues, the expression of FDX1 in 19 adjacent tissues was higher than in cancer tissues. In addition, the expression level of FDX1 in adjacent nontumor tissues was significantly higher than in tumor tissues (*P* < 0.05) (Figure 2(a)). WB analysis showed that in 16 pairs of ccRCC tissues, FDX1 expression was significantly higher in tumor-adjacent tissues than in tumor tissues (Figure 2(b)). Immunohistochemical results showed that in 5 pairs of ccRCC tissues, FDX1 was positive in tumor-adjacent tissues while negative in tumor tissues (Figure 3(c)).

### 3.4. High Expression of FDX1 in ccRCC Was Related to Well Overall Survival

Compared with patients with low expression of FDX1, patients with high FDX1 were significantly associated with a good overall survival (OS) rate (*P* < 0.05, Figure 1(d)). The same results were shown in the relationship between FDX1 expression and the progression-free survival or disease-specific survival of ccRCC patients based on TCGA (Figures 1(e) and 3(f)).

### 3.5. The Relationship between FDX1 Expression and Clinicopathological Parameters

The samples with missing clinical data were deleted.  Table 3 summarizes the correlation between the expression levels of FDX1 in ccRCC patients with various clinicopathological parameters. In addition, the expression level of FDX1 was different in groups classified based on the pathological grade, gender, TNM stage, T stage, lymph node metastasis, and distant metastasis (*P* < 0.05) (Figure 3).

### 3.6. The Effect of FDX1 Expression on Survival Based on Univariate and Multivariate Analysis

The samples with missing clinical data were deleted. Univariate and multivariate analyses were performed in ccRCC patients based on Cox proportional risk regression models to assess the effect of FDX1 expression and other clinical pathology factors on survival. Univariate analysis showed that age, pathological grade, TNM stage, T classification, lymph node metastasis, distant metastasis, and FDX1 expression were important predictors of survival (Table 4). In addition, the multivariate analysis showed that the FDX1 high expression was an important independent predictor of overall survival (Table 4 and Figure 4(a)).

### 3.7. Expression of FDX1 Protein in ccRCC and Normal Kidney Tissues

Using the HPA database, FDX1 immunohistochemical antibody (Antibody HPA062087) was used. Immunohistochemical results of normal kidney tissue and ccRCC tissue were analyzed.  Figure 2(d) shows that antibody staining occurred in renal tubular cells in normal kidney tissue. The expression of FDX1 protein in normal kidney tissue was further confirmed.

### 3.8. FDX1-Interacting Protein Network

The input was done according to the aforementioned conditions to obtain Figure 4(b). Among them, CYCS, AKR1B1, CYP11A1, FDXR, NFS1, LYRM4, ISCU, FXN, LIAS, LIPT2, and LIPT1 interacted with FDX1 in the PPI network. Additionally, LIAS and LIPT1 genes are involved in the regulation of cuprotosis. The high expression of LIPT1 and LIAS in ccRCC was related to overall survival (Figures 4(c) and 4(d)).

### 3.9. FDX1-Related Signaling Pathways by GSEA

GSEA algorithm analysis showed that beta-alanine metabolism, biosynthesis of unsaturated fatty acids, butanoate metabolism, citrate cycle, TCA cycle, complement, and coagulation cascades were enriched differently in the high expression of FDX1. The expression of FDX1 inhibits adherens junction, base excision repair, cell cycle, cytosolic DNA sensing pathway, and DNA replication pathway (Figure 4(e)). According to the ssGSEA algorithm, the low expression of FDX1 was related to tumor proliferation signature and DNA replication pathway (*P* < 0.05) (Figure 4(f)).

### 3.10. Analysis of FDX1 in Pan-Cancer

The results showed that the high expression of FDX1 was a good prognostic factor in some cancers (HR < 1), stomach adenocarcinoma (STAD), rectum adenocarcinoma (READ), liver hepatocellular carcinoma (LIHC), cervical squamous cell carcinoma (CSCC), bladder urothelial carcinoma (BLCA), kidney chromophobe (KICH), kidney renal papillary cell carcinoma (KIRP), cholangiocarcinoma (CHOL), mesothelioma (MESO), pheochromocytoma and paraganglioma (PCPG), and uterine carcinosarcoma (UCS) (Figures 5(a) and 5(b)). At the same time, FDX1 was highly expressed in the adjacent tissues (Figure 5(c)).

## 4. Discussion

According to the pathological features, renal cell carcinoma can be divided into clear cell carcinoma, papillary renal cell carcinoma, chromophobe renal cell carcinoma, and Bellini collecting duct carcinoma. Among all the types, clear cell carcinoma is the most common [14]. Many renal cancers are resistant to chemotherapy and radiotherapy [15]. Therefore, regulatory cell death is an ideal treatment strategy for renal cell carcinoma, which may overcome the drug resistance in renal cell carcinoma [16]. Yang et al. tested the sensitivity of 117 tumor cell lines for ferroptosis caused by erastin. They found that the diffuse large B cell lymphoma and renal cell carcinoma were particularly sensitive to iron death regulated by GPX4 [17]. Miess et al. found that GPX3 and GPX4 were lethal to renal clear cell carcinoma. Further, they have shown that by blocking the GSH synthesis, renal clear cell carcinoma became more sensitive to iron death, thus inhibiting tumor growth. In renal cancer cells lacking the VHL gene, the newly expressed VHL produced resistance to iron death [18]. The concept of cuprotosis was first proposed in a paper published on Science on 17 March 2022 [11]. Copper-dependent controlled cell death is a new pathway different from the known cell death mechanism. However, cuprotosis effect on the progress of tumors like ferroptosis is not yet known. The FDX1 gene was essential for copper-induced cell death [11]. FDX1 is an upstream regulator of protein lipoylation. Thus, we studied the FDX1 expression in ccRCC and analyzed its effect on the prognosis of patients.

In this study, we determined if the expression of FDX1 played a role in the progression of ccRCC, especially as a prognostic factor. Firstly, we analyzed the RNA-seq data in TCGA database and compared the expression of FDX1 in ccRCC and adjacent nontumor tissues. The expression level of FDX1 mRNA in adjacent nontumor tissues was significantly higher than that in tumor tissues. Further, we verified the expression difference of FDX1 by GEO data. To verify the difference in FDX1 expression in TCGA and GEO database, we used qRT-PCR, WB, and IHC. All results showed that the FDX1 in adjacent nontumor tissues was significantly higher than that in tumor tissues. In addition, the expression level of FDX1 was different in groups classified according to pathological grade, gender, TNM stage, T stage, lymph node metastasis, and distant metastasis (*P* < 0.05). Furthermore, the relationship between FDX1 expression and clinicopathological parameters was analyzed. Kaplan-Meier survival analysis revealed that the prognosis of the high FDX1 expression group was better than the low FDX1 expression group. Univariate analysis showed that high FDX1 expression was associated with better OS. Other clinicopathological parameters including age, pathological grade, TNM stage, T stage, lymph node metastasis, and distant metastasis were related to the prognosis of ccRCC patients. Importantly, FXD1 was an independent prognostic factor for the overall survival in ccRCC patients and proved its potential as a biomarker of ccRCC. Immunohistochemical analysis of the HPA database confirmed the expression of FDX1 protein in normal kidney and renal tubular tissue. Renal cell carcinoma clear cell type comes from renal tubular cells, and its immunophenotype is closer to proximal convoluted tubule epithelium (expressing Vimentin and CD10) [19]. Ferredoxin reductase (FDXR) interacts with FDX1D protein, which is a target of p53. It modulates p53-dependent apoptosis necessary for steroidogenesis and biogenesis of iron-sulfur clusters [20].

Based on TCGA data, we explored FDX1-related signal transduction pathway through GSEA. Our results demonstrate that ccRCC patients with high FDX1 expression may inhibit the adherens junction, base excision repair, cell cycle, cytosolic DNA sensing pathway, and DNA replication pathway. These are closely related to the early onset of cancer along with the risk of tumor progression and metastasis [21–23]. The abnormality of the cell cycle process is one of the basic mechanisms of tumorigenesis. It makes the regulator of the cell cycle mechanism a reasonable target for anticancer therapy [24]. The high expression of FDX1 may inhibit the expression of cell cycle key proteins, thereby inhibiting tumor progression. These new biological processes identified by GSEA helped us to gain a better knowledge of molecular mechanisms existing in ccRCC. However, these FDX1-enriched pathways will be validated in future experiments. According to the ssGSEA algorithm, the low expression was related to tumor proliferation signature and DNA replication pathway. Pan-cancer analysis showed that the high expression of FDX1 served as a good prognostic factor in some cancers (HR < 1). These results indicate that the FDX1 may be a tumor suppressor gene and play a vital role in the progress of ccRCC.

Ferredoxin is a low molecular weight protein with a negative charge at neutral pH. It contains iron-sulfur clusters as redox-active groups [25]. Humans possess two mitochondrial ferredoxins, ferredoxin 1 (FDX1) and ferredoxin 2 (FDX2). These ferredoxins have distinct roles in steroidogenesis, heme, and Fe/S cluster biosynthesis [26]. FDX1 encodes a small ferritin protein, which transfers electrons from NADPH to mitochondrial cytochrome P450 through ferredoxin reductase and participates in the steroid, vitamin D, and bile acid metabolism. Shi et al. suggest that interfering with FDX1 can disrupt iron-sulfur cluster assembly. Thus, it is important for maintaining normal cytosolic and mitochondrial iron homeostasis [27]. Wang et al. performed unique identifier technically labeled transcriptomics on granulosa cells of PCOS and control group women to extract key genes. They found that FDX1 was related to steroid metabolism in mitochondria and may be involved in developing polycystic ovary syndrome [28]. However, there are few research on the role of FDX1 expression in various cancers. Further, Zhang et al. found a poor prognosis in lung adenocarcinoma patients with low expression of FDX1 [29].

Previous studies have shown that the FDX1 encodes a reductase known to reduce Cu2^+^ to its more toxic form, Cu1^+^, which is a direct target of elesclomol [30]. Despite blocking the known cell death modes (such as apoptosis and ferroptosis), the cells treated with copper carriers still died. The research team coined this new way of cell death as cuprotosis [30]. The research team blocks the known cell death modes (such as apoptosis and ferroptosis), and the cells treated with copper carriers will still die. The research team thinks that this is a new way of cell death and named it cuprotosis [11]. The research team used CRISPR screening to identify several key genes that promote the death of copper, including the FDX1 gene encoding the target protein of elesclomol [11]. FDX1 is an upstream regulator of protein lipoylation. In this study, the STRING database showed that LIAS and LIPT1 interact with FDX1 in the PPI network, which are also involved in the regulation of cuprotosis. LIPT1 encodes components of the lipoic acid pathway [11]. Of note, the high expression of LIPT1 and LIAS in ccRCC was related to the overall survival response. Though our study had some limitations, the overall results indicate that copper death may play a role in the occurrence and development of ccRCC. However, the cuprotosis regulatory role in ccRCC needs further verification.

Copper ion carrier drugs such as elesclomol (ES), disulfiram, and NSC319726 can induce cell death [31, 32]. ES has been reported to have considerable anticancer activity, but the underlying mechanism remains unclear [33]. Gao et al. found that ES-induced copper chelation inhibits colorectal cancer by targeting ATP7A. In our future experiments, copper ionophore drugs will be used to stimulate ccRCC cells with high expression of FDX1 to assess the induction of cuprotosis. Various copper ionophores are used to induce copper death. Its potential molecular mechanism suggests that copper ionophores can kill ccRCC cells (with high expression of FDX1), which may become a new direction of tumor therapy with important clinical guiding significance.

## 5. Conclusions

Our research first analyzed TCGA database and found that the expression of cuprotosis-related gene FDX1 in adjacent nontumor tissues was higher than that in tumor tissues. At the same time, the expression difference of FDX1 was verified by a variety of experimental methods Furthermore, the expression of FDX1 has closely related to the clinicopathological features, occurrence, and development of ccRCC. Importantly, univariate and multivariate survival analysis confirmed that the increased expression of FDX1 was an independent prognostic factor for prolonged OS in ccRCC patients. However, cuprotosis involvement in the occurrence and development of ccRCC disease needs further investigations.

## Figures and Tables

**Figure 1:** The expression of FDX1 based on TCGA data (a). The expression of FDX1 based on GEO data (GSE53757) (b). The expression of FDX1 based on GEO data (GSE40435) (c). The relationship between FDX1 expression and the overall survival of ccRCC patients based on TCGA (d). The relationship between FDX1 expression and the progression-free survival of ccRCC patients based on TCGA (e). The relationship between FDX1 expression and the disease-specific survival of ccRCC patients based on TCGA (f). ^∗^*P* < 0.05, ^∗∗^*P* < 0.01, and ^∗∗∗^*P* < 0.001.

**Figure 2:** qRT-PCR shows differential expression of FDX1 in adjacent nontumor tissues and tumor tissues (a). WB shows differential expression of FDX1 in adjacent nontumor tissues and tumor tissues (b). FDX1 protein was positive in adjacent nontumor tissues and negative in ccRCC tissues (IHC, 200x) (c). FDX1 protein was positive in normal kidney tissue and negative in ccRCC tissues based on HPA database (IHC, 200x) (d). ^∗^*P* < 0.05, ^∗∗^*P* < 0.01, and ^∗∗∗^*P* < 0.001.

**Figure 3:** The expression of FDX1 was grouped by (a) pathological stage, (b) gender, (c) ages, (d) TNM stage, (e) T stage, (f) lymph node metastasis, and (g) distant metastasis. ^∗^*P* < 0.05, ^∗∗^*P* < 0.01, and ^∗∗∗^*P* < 0.001.

**Figure 4:** Forest plot for the multivariate Cox proportional hazard regression model. FDX1 was an independent predictor of well survival rate (a). The network diagram of FDX1-related protein (b). The relationship between LIPT1 expression and the prognosis of ccRCC patients based on TCGA (c). The relationship between LIAS expression and the prognosis of ccRCC patients based on TCGA (d). A merged enrichment plot from gene set enrichment analysis (e). According to ssGSEA algorithm, the relationship between the expression of FDX1 and different pathway (f). ^∗^*P* < 0.05, ^∗∗^*P* < 0.01, and ^∗∗∗^*P* < 0.001.

**Figure 5:** The relationship between FDX1 expression and the prognosis of multiple tumors based on TCGA (a). The *P* value, risk coefficient (HR), and confidence interval of a gene in multiple tumors were analyzed by univariate Cox regression (b). FDX1 expression in normal and tumor tissues based on TCGA (c). ^∗^*P* < 0.05, ^∗∗^*P* < 0.01, and ^∗∗∗^*P* < 0.001.

**Table 1:** Information of selected TCGA data.

Characteristics	*N*	Percentages
Gender		
Male	344	64.9%
Female	186	35.1%
Age		
<60 years	245	47.9%
>60 years	266	52.1%
TNM		
I-II stage	322	61.1%
III-IV stage	205	38.9%
Tumor		
T1	271	54.4%
T2	55	11.0%
T3	172	34.5%
Lymph node metastasis		
Negative	239	93.7%
Positive	16	6.3%
Distant metastasis		
Negative	440	84.6%
Positive	80	15.4%
Grade		
I-II	241	46.2%
III-IV	281	53.8%
Vital status		
Death	173	32.6%
Alive	357	67.4%

**Table 2:** Information of selected GEO data.

GEO data	Country	Year	Platform	Sample	*n*
GSE53757	USA	2014	GPL570	Adjacent nontumor tissue	72
				Tumor tissue	72
GSE40435	France	2013	GPL10558	Adjacent nontumor tissue	101
				Tumor tissue	101

**Table 3:** Relationships between FDX1 expression and clinicopathological parameters in ccRCC.

Clinicopathological parameters	FDX1 expression			
	High	Low	Total	*P* value
Gender				0.045
Male	183 (53.2%)	161 (46.8%)	344	
Female	82 (44.1%)	104 (55.9%)	186	
Age				0.422
<60 years	124 (50.6%)	121 (49.4%)	245	
>60 years	138 (51.9%)	128 (48.1%)	266	
TNM				0.015
I-II stage	174 (54.0%)	148 (46.0%)	322	
III-IV stage	90 (43.9%)	115 (56.1%)	205	
Tumor				0.025
T1	147 (54.2%)	124 (45.8%)	271	
T3	76 (44.2%)	96 (55.8%)	172	
Lymph node metastasis				0.008
Negative	125 (52.3%)	114 (47.7%)	239	
Positive	3 (18.8%)	13 (81.3%)	16	
Distant metastasis				0.085
Negative	227 (51.6%)	213 (48.8%)	440	
Positive	34 (42.5%)	46 (57.5%)	80	
Grade				0.005
I-II	136 (56.4%)	105 (43.6%)	241	
III-IV	126 (44.8%)	155 (55.2%)	281	

**Table 4:** Univariate analysis and multivariate analysis of the correlation of FDX1 expression with OS among ccRCC patients.

Parameter	Univariate analysis			Multivariate analysis		
	HR	95% CI	*P* value	HR	95% CI	*P* value
Age	1.023	1.005-1.041	0.010	1.036	1.016-1.056	<0.001
Gender	0.975	0.642-1.481	0.907			
Pathological grade	2.199	1.653-2.925	<0.001	1.473	1.058-2.052	0.022
Stage	1.837	1.522-2.216	<0.001			
T classification	1.909	1.514-2.407	<0.001			
M classification	4.032	2.610-6.229	<0.001			
N classification	2.909	1.505-5.621	0.001			
FDX1	0.507	0.318-0.807	0.004	0.529	0.343-0.817	0.004

## Data Availability

All research data are from TCGA database and GEO database, which have been marked in the text. Original pictures can be provided if readers have reasonable requests.

## References

[1] Bray F., Ferlay J., Soerjomataram I., Siegel R. L., Torre L. A., Jemal A. (2018). Global cancer statistics 2018: GLOBOCAN estimates of incidence and mortality worldwide for 36 cancers in 185 countries. *CA: A Cancer Journal for Clinicians*.

[2] Jonasch E., Gao J., Rathmell W. K. (2014). Renal cell carcinoma. *BMJ*.

[3] Unverzagt S., Moldenhauer I., Nothacker M. (2017). Immunotherapy for metastatic renal cell carcinoma. *Cochrane Database of Systematic Reviews*.

[4] Kroemer G., el-Deiry W. S., Golstein P. (2005). Classification of cell death: recommendations of the Nomenclature Committee on Cell Death. *Cell Death and Differentiation*.

[5] Dixon S. J., Lemberg K. M., Lamprecht M. R. (2012). Ferroptosis: an iron-dependent form of nonapoptotic cell death. *Cell*.

[6] Jiang X., Stockwell B. R., Conrad M. (2021). Ferroptosis: mechanisms, biology and role in disease. *Nature Reviews Molecular Cell Biology*.

[7] Ding Y., Chen X., Liu C. (2021). Identification of a small molecule as inducer of ferroptosis and apoptosis through ubiquitination of GPX4 in triple negative breast cancer cells. *Journal of Hematology & Oncology*.

[8] Xu S., He Y., Lin L., Chen P., Chen M., Zhang S. (2021). The emerging role of ferroptosis in intestinal disease. *Cell Death & Disease*.

[9] Wu Y., Zhang S., Gong X. (2020). The epigenetic regulators and metabolic changes in ferroptosis-associated cancer progression. *Molecular Cancer*.

[10] Singh D. (2021). Current updates and future perspectives on the management of renal cell carcinoma. *Life Sciences*.

[11] Tsvetkov P., Coy S., Petrova B. (2022). Copper induces cell death by targeting lipoylated TCA cycle proteins. *Science*.

[12] Wei J., Huang K., Chen Z. (2020). Characterization of glycolysis-associated molecules in the tumor microenvironment revealed by pan-cancer tissues and lung cancer single cell data. *Cancers*.

[13] Chen X., Li X., Hu X. (2020). LUM expression and its prognostic significance in gastric cancer. *Frontiers in Oncology*.

[14] Delahunt B., Eble J. N., Egevad L., Samaratunga H. (2019). Grading of renal cell carcinoma. *Histopathology*.

[15] Barata P. C., Rini B. I. (2017). Treatment of renal cell carcinoma: current status and future directions. *CA: A Cancer Journal for Clinicians*.

[16] Xu W., Atkins M. B., Mcdermott D. F. (2020). Checkpoint inhibitor immunotherapy in kidney cancer. *Nature Reviews. Urology*.

[17] Yang W. S., SriRamaratnam R., Welsch M. E. (2014). Regulation of ferroptotic cancer cell death by GPX4. *Cell*.

[18] Miess H., Dankworth B., Gouw A. M. (2018). The glutathione redox system is essential to prevent ferroptosis caused by impaired lipid metabolism in clear cell renal cell carcinoma. *Oncogene*.

[19] Truong L. D., Shen S. S. (2011). Immunohistochemical diagnosis of renal neoplasms. *Archives of Pathology & Laboratory Medicine*.

[20] Zhang Y., Qian Y., Zhang J. (2017). Ferredoxin reductase is critical for p53-dependent tumor suppression via iron regulatory protein 2. *Genes & Development*.

[21] Dalton S. (2015). Linking the cell cycle to cell fate decisions. *Trends in Cell Biology*.

[22] Shen J. Z., Qiu Z., Wu Q. (2021). FBXO44 promotes DNA replication-coupled repetitive element silencing in cancer cells. *Cell*.

[23] Kwon J., Bakhoum S. F. (2020). The cytosolic DNA-sensing cGAS-STING pathway in cancer. *Cancer Discovery*.

[24] Icard P., Fournel L., Wu Z., Alifano M., Lincet H. (2019). Interconnection between metabolism and cell cycle in cancer. *Trends in Biochemical Sciences*.

[25] Grinberg A. V., Hannemann F., Schiffler B., Müller J., Heinemann U., Bernhardt R. (2000). Adrenodoxin: structure, stability, and electron transfer properties. *Proteins*.

[26] Sheftel A. D., Stehling O., Pierik A. J. (2010). Humans possess two mitochondrial ferredoxins, Fdx1 and Fdx2, with distinct roles in steroidogenesis, heme, and Fe/S cluster biosynthesis. *Proceedings of the National Academy of Sciences of the United States of America*.

[27] Shi Y., Ghosh M., Kovtunovych G., Crooks D. R., Rouault T. A. (2012). Both human ferredoxins 1 and 2 and ferredoxin reductase are important for iron-sulfur cluster biogenesis. *Biochimica et Biophysica Acta*.

[28] Wang Z., Dong H., Yang L., Yi P., Wang Q., Huang D. (2021). The role of FDX1 in granulosa cell of polycystic ovary syndrome (PCOS). *BMC Endocrine Disorders*.

[29] Zhang Z., Ma Y., Guo X. (2021). FDX1 can impact the prognosis and mediate the metabolism of lung adenocarcinoma. *Frontiers in Pharmacology*.

[30] Tsvetkov P., Detappe A., Cai K. (2019). Mitochondrial metabolism promotes adaptation to proteotoxic stress. *Nature Chemical Biology*.

[31] Viola-Rhenals M., Patel K. R., Jaimes-Santamaria L., Wu G., Liu J., Dou Q. P. (2018). Recent advances in Antabuse (disulfiram): the importance of its metal-binding ability to its anticancer activity. *Current Medicinal Chemistry*.

[32] Shimada K., Reznik E., Stokes M. E. (2018). Copper-binding small molecule induces oxidative stress and cell-cycle arrest in glioblastoma-patient-derived cells. *Cell Chemical Biology*.

[33] Gao W., Huang Z., Duan J., Nice E. C., Lin J., Huang C. (2021). Elesclomol induces copper-dependent ferroptosis in colorectal cancer cells via degradation of ATP7A. *Molecular Oncology*.

